# Drone Assisted Robust Emergency Service Management for Elderly Chronic Disease

**DOI:** 10.1155/2021/5552350

**Published:** 2021-04-09

**Authors:** Shengqiang Jiang, Yong Jin, Kaijian Xia

**Affiliations:** ^1^Department of Science and Technology, Nanjing Medical University, Nanjing, Jiangsu, China; ^2^School of Computer Science and Engineering, Changshu Institute of Technology, Changshu, Jiangsu, China; ^3^The Affiliated Changshu Hospital of Soochow University (Changshu No. 1 People's Hospital), Changshu, Jiangsu, China

## Abstract

It is important to monitor the early screening of chronic diseases, predict the risk, and provide the comprehensive management of chronic diseases for the elderly. However, it is difficult to provide the robust and real-time emergency service for elderly chronic disease because of the complex social network and diversity of elderly chronic disease service. To address these issues, we design a new drone assisted robust emergency service system. We formulate the Drone assisted Management (DM) problem to minimize the total time cost of drone subject to all elderly chronic disease services which can be guaranteed exactly once by the drone under its energy constraint. Then, we propose the DRS algorithm to solve the DM problem. To provide the robust and real-time service, we further formulate the Charging driven Drone assisted Management (CDM) problem and present the CDRS algorithm to solve the CDM problem. Through the theoretical analysis and numerical simulation experiments, we demonstrate that DRS and CDRS can decrease the total time cost by 37.61% and increase the QoE by 112.80% through the designed system, respectively.

## 1. Introduction

The HelpAge International has released the report of the global aging business observation index 2015 [1]. According to the report, there are about 901 million people aged 60 and above, accounting for 12.3% of the world's population. By 2030, this proportion will reach 16.5%. Globally, the number of people over the age of 60 exceeds the number of children below 5 years of age. By 2050, the number of people over 60 will exceed the number of people below 15 years of age. According to the report, China has the largest aging population in the world, with 209 million. By 2025, the total number of China's elderly population will be nearly 300 million. By 2035, there will be 400 million elderly people in China; that is, one in every three people is an elderly person. In the past 20 years, the proportion of the aging population has increased from 20% to 30%, and the development is very rapid [2].

The World Health Organization (WHO) reported that 63% of all deaths globally are due to chronic diseases, such as cardiovascular diseases, diabetes, cancers, and chronic respiratory illnesses. The care of elderly may involve multiple healthcare professionals in different locations, as well as a variety of medications and treatments. Thus, good management and a proactive approach to diagnosis and treatment are important [3]. Therefore, chronic noncommunicable diseases and their risk factors are regularly detected, continuously monitored, evaluated, and comprehensively intervened. The main contents include early screening of chronic diseases, risk prediction of chronic diseases, early warning and comprehensive intervention, and comprehensive service management of chronic diseases. The evaluation of chronic disease service management effect is particularly important.

However, chronic disease service management faces many difficulties. First of all, the doctor centered chronic disease service results in resource mismatch and lack of personalized service. Secondly, the core of chronic disease service management is user education and follow-up supervision or incentive mechanism, which is difficult to adapt to the particularity of elderly patients. It is necessary to integrate hospitals, communities, and families to improve the real-time performance of chronic disease service management, with poor robustness and reliability.

Fortunately, drones have performed well in many service areas. Kim et al. [4] addressed the drone-aided delivery and pickup planning of medication and test kits for patients with chronic diseases who are required to visit clinics for routine health examinations and/or refill medicine in rural areas. Nenni et al. [5] redesigned the entire Emergency Medical Services model by including drones. Radosveta et al. [6] introduced some of the most recent and interesting applications that drones can find in creating ambient assisted living environments for the elderly.

However, the battery of drone is limited, so it is necessary to solve the dual constraints of scheduling ground charging stations and the demand of elderly chronic disease management. The existing research mainly focuses on how to improve the chronic disease service level of drone, but there is little research on how to improve the service cycle, efficiency, effect, and the robustness of elderly chronic disease emergency service. We designed a drone assisted elderly chronic disease management system, as shown in Figure 1. When the elderly are in the outdoor shopping center, train station, park, bus stops, apartment, suburban house, city house, and stadium, the drones can carry the drugs and emergency medical supplies and have the capacity to carry modest payloads and can transport them quickly to their destination in case of sudden chronic disease when the real-time emergency service is needed.

However, in the above scenario, we face many challenges. First of all, the energy of drone is limited, and a flight can serve the elderly and the service time is limited. How to provide the most effective service for the elderly in the limited time makes it very difficult to optimize the drone scheduling and chronic disease resource matching. When the residual energy of drone is insufficient, it needs to go to the charging stations deployed on ground or roof to replenish energy. Secondly, there is a time conflict between drone charging scheduling and the robustness of chronic disease emergency service management. It is very difficult to consider charging demand and robust service simultaneously in drone scheduling.

Our key contributions can be summarized as follows:

- We design a new drone assisted robust emergency service system through the drone assistance.
- We formulate the problem of Drone assisted Management (DM) to minimize the total time cost of drone subject to all elderly chronic disease services which can be guaranteed exactly once by the drone under its energy constraint and propose the Drone assisted Robust emergency Service (DRS) algorithm to solve the DM problem.
- Considering the guarantee of robustness and real time of emergency service for elderly chronic disease, we further formulate the Charging driven Drone assisted Management (CDM) problem to maximize the service utility and we present an algorithm to solve the CDM problem.
- We conduct extensive simulations for the designed system and proposed algorithms. The results show that the DRS algorithm and CDRS algorithm can decrease the total time cost by 37.61% and increase the Quality of Experience (QoE) by 112.80% through the designed system, respectively.

The rest of the paper is organized as follows. We review the state-of-the-art research in Section 2. We present the system model and formulate the CDM problem in Section 3. We formulate the DM problem and propose the corresponding algorithm in Section 4. We design the algorithm for solving CDM problem in Section 5. We conduct the simulations in Section 6, respectively. We conclude this work in Section 7.

## 2. Related Work

The current situation of chronic disease management in the elderly is discussed as follows. Lima et al. [7] studied the impact of chronic disease and the number of diseases on the various aspects of health-related quality of life among the elderly in São Paulo, Brazil. Lawlor et al. [8] researched the associations between having had a fall and chronic diseases and drug use in elderly women. Rocha and Ciosak [9] found that the changes brought about the diagnosis of chronic disease and its implications for the adaptation to the new way of life. The management of these changes is complex, and many factors influence positively and negatively.

About the status of drone service, Cheskes et al. [10] examined the feasibility of a novel Automated External Defibrillators (AED) drone delivery method for rural and remote sudden cardiac arrest and showed that the AED drone is feasible with the potential for improvements in response time during simulated sudden cardiac arrest scenarios. Angurala et al. [11] used the drone service to reduce the risk of infection to the doctors or other medical staff, thereby preventing the disease spread. Hart et al. [12] studied the acceptability and perceived utility of Unmanned Aerial Vehicle (UAV) technology to Mass Casualty Incidents (MCI) scene management.

About the drone scheduling, Boysen et al. [13] designed a drone schedule to minimize the total duration of the delivery tour subject to supplying all customers under considering a fixed sequence of stops constituting a truck route and a set of customers to be supplied. Kim et al. [14] proposed a robust optimization approach to find the optimal flight schedule including the number of drones and flight paths in the flight network considering uncertain battery duration. Wang et al. [15] proposed a novel routing and scheduling algorithm, referred to as hybrid truck-drone delivery algorithm, to solve the hybrid parcel delivery problem.

About the charging scheme of drone, Hu et al. [16] proposed a fully automatic charging station which operates wirelessly. Raciti et al. [17] proposed a current tuning mechanism that compensates for this variability in a single-inverter multipad charging station. Kim et al. [18] proposed a cloud-based drone navigation system for efficient drone battery charging in drone networks.

The system we designed is different from the above research. Our system integrates the ground charging stations and the elderly points that need emergency chronic disease services. In particular, we consider the charging efficiency of drone, the real-time response of emergency chronic disease service, and the emergency service management robustness of the elderly chronic disease all together. We solved two problems. The first problem maximizes the management utility of drone to the elderly chronic disease emergency service without considering the charging. In order to expand the scope of drone service and improve the emergency service management robustness of elderly chronic disease, the second problem consider the drone charging and the elderly chronic disease emergency service requirements.

## 3. Energy Constrained Drone Assisted Management

### 3.1. System Model and Problem Formulation

We consider the living quarters for the elderly, including the outdoor shopping center, train station, park, bus stops, apartment, suburban house, city house, and stadium. The locations of these venues are known and fixed. We define them as emergency service points. There is a drone in the area to provide emergency services for chronic diseases. The elderly people may make the chronic disease emergency service requests for cardiovascular diseases, diabetes, cancers, and chronic respiratory illnesses at any time in the living area.

Firstly, the distance between any two emergency service points in the living area is less than the maximum flight distance of drone. Therefore, drone can provide relevant medical services for multiple emergency service points without charging. Secondly, the elderly are not in a completely helpless state; that is, they can simply interact with drone and save themselves. Therefore, the emergency service of drone can be completed in a short time. Then, the impact of external natural environment such as wind and complex environment of buildings on drone flight energy consumption and time is not considered. Therefore, the drone always keeps constant speed. Flight time and energy consumption are only related to traveling distance. Finally, we assume that the charging stations deployed on the ground or roof can satisfy the charging requirements of drone at any time.

Without loss of generality, let *o* be the set of *n* elderly people and let *r*_i_ be the time cost of emergency service for the *i*-th elderly chronic disease service. Let *S* be the set of *m* charging stations and let *φ* be the charging power of charging station. Note that the charging power of each charging station is the same. Let *ν*, *σ*_*h*_, *σ*_*f*_, and *C*_max_ be the flying speed, the unit hovering energy consumption, the unit flying energy consumption, and the battery capacity of drone, respectively. The drone is initially located at the depot, denoted by *d*_0_.

To formalize the emergency service management for elderly chronic disease, we use the undirected graph *G*=(*O* ∪ *S*, *E*) to represent the emergency service management network. *E* represents the set of service segments that connect the adjacent elderly people and/or charging station. The weight on any edge *e* ∈ *E* is time cost *t*_*e*_, which represents the consumed time when the drone passes through the edge *e*. Let *T* be the tour of drone and let *β* be the energy consumption of drone providing service for the elderly chronic disease. Let *c*_*e*_ be the energy consumption of drone passing through the edge *e*. In addition, let *𝒞*_*i*_ be the residual energy of drone after passing through the edge *e* and completing the *i*-th elderly chronic disease service. Let *T*_*i*_⊆*T* be the drone subtour from the depot to the *i*-th elderly chronic disease service. Let *τ*_*k*_  be the charging time for drone at charging station *s*_*k*_ ∈ *S*. We define the function *O*(*T*_*i*_) to indicate the elderly people serviced by the drone and *S*(*T*_*i*_) to indicate the charging stations visited by the drone in the tour *T*_*i*_, respectively. Let *c*_0_ be the initial energy of drone launching at *d*_0_. Then, *𝒞*_*i*_ can be calculated by the following equation:

(1) $$\begin{array}{c} C_{i}=c_{0}-\underset{e\in T_{i}}{\sum }c_{e}-\underset{o_{i^{\prime }}\in O\left(T_{i}\right)}{\sum }r_{i^{\prime }}\beta \;+\underset{s_{k}\in S\left(T_{i}\right)}{\sum }\tau_{k}\varphi . \end{array}$$

We define the service utility of the *i*-th elderly chronic disease service as function *f*(*o*_*i*_) listed as follows:

(2) $$\begin{array}{c} f\left(o_{i}\right)=\underset{n⟶\infty }{\lim}\frac{r_{i}}{\sum_{i\prime =1}^{i}r_{i^{\prime }}+\sum_{e\in T_{i}}t_{e}}. \end{array}$$

The objective of CDM is to design a drone tour starting from *d*_0_ to provide the chronic disease emergency service for the elderly exactly once to maximize the service utility under the energy constraint of drone. *x*_*i*,*j*_ is a binary variable to indicate whether the drone passes through the edge (*i*, *j*) ∈ *E*,  ∀ *o*_*i*_, *o*_*j*_ ∈ O. *x*_*i*,*j*_=1 if the drone passes through the edge (*i*, *j*) and *x*_*i*,*j*_=0 otherwise. The CDM problem can be formulated as follows:

(3) $$\begin{array}{c} \text{CDM }\max\overset{n}{\underset{i=1}{\sum }}\overset{n}{\underset{j=1}{\sum }}x_{i,j}\underset{o_{j}\in O}{\sum }f\left(o_{j}\right)\\ \text{s.t.}\\ \left(\text{a}\right)x_{i,j}\in \left\{0,1\right\},\;\forall o_{i},\;o_{j}\in O\\ \left(\text{b}\right)\overset{n}{\underset{i=1}{\sum }}x_{i,j}=1,\;\forall o_{j}\in O\\ \left(\text{c}\right)\overset{n}{\underset{j=1}{\sum }}x_{i,j}=1,\;\forall o_{i}\in O\\ \left(\text{d}\right)c_{ij}+r_{i}\beta \;\leq C_{i},\forall o_{i},o_{i}\in O\left(T_{i}\right),T_{i}\subseteq T \end{array}$$

Constraint (a) gives the value range of *x*_*i*,*j*_. Constraints (b) and (c) ensure that each elderly chronic disease service is visited by the drone exactly once; that is, the drone can provide the corresponding elderly chronic disease service for all elderly people. Constraint (d) ensures that the sum of flying energy consumption of drone and providing the corresponding elderly chronic disease service is not larger than the residual energy of drone after visiting *o*_*i*_.

We listed the frequently used notations in Table 1.

## 4. Drone Assisted Management Scheme

### 4.1. Problem Formulation

Before solving the CDM problem, we first design the DM problem, which is formulated as follows:

(4) $$\begin{array}{c} \text{DM max}\overset{n}{\underset{i=1}{\sum }}\overset{n}{\underset{j=1}{\sum }}x_{i,j}\underset{o_{j}\in O}{\sum }f\left(o_{j}\right)\\ s\mathrm{.t}.\\ \left(\text{a}\right)x_{i,j}\in \left\{0,1\right\},\;\forall o_{i},o_{j}\in O\\ \left(\text{b}\right)\overset{n}{\underset{i=1}{\sum }}x_{i,j}=1,\;\forall o_{j}\in O\\ \left(\text{c}\right)\overset{n}{\underset{j=1}{\sum }}x_{i,j}=1,\;\forall o_{i}\in O\\ \left(\text{d}\right)\underset{e\in T}{\sum }c_{e}+\underset{o_{i}\in O}{\sum }r_{i}\beta \;\leq C_{\text{max}}. \end{array}$$

Constraint (d) ensures that the energy consumption sum of flying and elderly chronic disease service is not larger than the battery capacity of drone.

From the primal dual theory, we define the Dual DM (DDM) problem listed in the following equation:

(5) $$\begin{array}{c} \text{DDM}\min\underset{e\in T}{\sum }c_{e}+\underset{o_{i}\in O}{\sum }r_{i}\beta \;\\ s.t.\\ \left(\text{a}\right)x_{i,j}\in \left\{0,1\right\},\;\forall o_{i},o_{j}\in O\\ \left(\text{b}\right)\overset{n}{\underset{i=1}{\sum }}x_{i,j}=1,\;\forall o_{j}\in O\\ \left(\text{c}\right)\overset{n}{\underset{j=1}{\sum }}x_{i,j}=1,\;\forall o_{i}\in O\\ \left(d\right)\overset{n}{\underset{i=1}{\sum }}\overset{n}{\underset{j=1}{\sum }}x_{i,j}\underset{o_{j}\in O}{\sum }f\left(o_{j}\right)\geq \rho . \end{array}$$

Constraint (d) ensures that the utility of elderly chronic disease service is not less than *ρ*, where *ρ* indicates the lower bound of quality of elderly chronic disease service.

### 4.2. Algorithm Design and Analysis

The objective of DDM problem is to find a drone tour to provide the elderly chronic disease service for all elderly people with minimum energy consumption under the constraint of energy of drone. Note that the solution for the DDM problem is the solution for the DM problem following Theorem 1.

**Theorem 1 .**

DM problem is equivalent to the DDM problem.

Clearly, the DDM problem is NP-hard to find the optimal tour for the drone from the following theorem.

**Theorem 2 .**

DM problem is NP-hard.

**Proof**

The problem is to visit all elderly people on the route of drone exactly once and return the depot with the minimum energy cost. This problem is a Traveling Salesman Problem (TSP) actually. Since the TSP is a well-known NP-hard problem, the DM problem is NP-hard.

Moreover, we design the Drone assisted Robust emergency Service (DRS) algorithm to solve the DM problem. The basic idea is given as follows: First, we used the primal dual algorithm for minimum weight vertex-covering problem to finish the transformation equivalently from the DM problem to the DDM problem [19]. Second, we solve a TSP following the NITSP algorithm [20]. The above process is illustrated in Algorithm 1.

There are five steps in Algorithm 1, which are listed as follows:

  Step 1: Construct the graph *G* according to the set of *O* (Line 1);
  Step 2: Construct the dual linear programming problem (Line 2);
  Step 3: Update *y*_*i*,*k*_ when there exists an edge satisfying the conditions in Line 6;
  Step 4: Initialize the set *z*_*i*_,  *i*=1,2,…, *n* (Lines 8–12);
  Step 5: Find the tour *T* through NITSP based on {*z*_*i*_*|* *i*=1,2,…, *n*} (Line 13).

**Theorem 3 .**

DRS is a polynomial-time approximation algorithm for DM problem.

**Proof**

The running time of Lines 1–12 is *O*(*n*^3.5^). The running time of Line 13 is polynomial.

Let opt denote the optimal solution of the DM problem. Let ${\tilde{y}}_{i,j}$ be the final solution of Lines 1–12 for each edge (*i*, *j*) ∈ *E*, *i* ≠ *j*. From Lines 5–7, there is at least one vertex *o*_*i*_ of edge (*i*, *j*) ∈ *E*, which satisfies the following equation:

(6) $$\begin{array}{c} \sum_{j:\left(i,j\right)\in E}y_{i,j}=\rho_{i} \end{array}$$

Hence, each edge (*i*, *j*) ∈ *E* is covered by the set ℛ.

We found that ${\left({\tilde{y}}_{i,j}\right)}_{\left(i,j\right)\in E}$ is a dual feasible solution for the primal dual linear programming problem, that is, DDM problem. So, we have

(7) $$\begin{array}{c} \underset{j:\left(i,j\right)\in E}{\sum }{\tilde{y}}_{i,j}\leq \text{opt}. \end{array}$$

Note that, for each *i*=1,2,…, *n*, we have

(8) $$\begin{array}{c} {\bar{z}}_{i}=1\text{ if and only if }\underset{j:\left(i,j\right)\in E}{\sum }y_{i,j}=\rho_{i}. \end{array}$$

Therefore, we have

(9) $$\begin{array}{c} \overset{n}{\underset{i=1}{\sum }}\rho_{i}{\bar{z}}_{i}=\underset{{\bar{z}}_{i}=1}{\sum }\rho_{i}\\ =\underset{{\bar{z}}_{i}=1}{\sum }\underset{\left(i,j\right)\in E}{\sum }{\tilde{y}}_{i,j}\\ \leq 2\underset{\left(i,j\right)\in E}{\sum }{\tilde{y}}_{i,j}\\ \leq 2\text{opt}. \end{array}$$

So, the process of Lines 1–12 can find an approximation solution for the DDM problem.

Finally, the NITSP algorithm can find an approximation solution for DM problem based on the set {*z*_*i*_*|* *i*=1,2,…, *n*}.

Above all, DRS is a polynomial-time approximation algorithm for solving the DM problem.

## 5. Charging Driven Drone Assisted Management

In this section, we present the Charging driven Drone assisted Robust emergency Service (CDRS) algorithm to solve the CDM problem. Obviously, the CDM problem is also NP-hard because the CDM problem is a tightened version of DM problem under considering the charging of drone. Hence, we have the following theorem.

**Theorem 4 .**

The CDM problem is NP-hard.

The basic idea of CDRS is illustrated as follows: we first complete the transformation from CDM problem to CDDM problem following primal dual theory, and we solve the CDDM problem through the solution of primal dual scheme for solving the generalized covering problem [21], and then we solve a TSP following the NITSP algorithm [20]. The above process is illustrated in Algorithm 2.

After primal dual theory, we define the CDDM problem listed in the following equation:

(10) $$\begin{array}{c} \text{CDDM}\min\;\underset{e\in T}{\sum }c_{e}+\underset{o_{i}\in O}{\sum }r_{i}\beta \;\\ s.t.\\ \left(\text{a}\right)x_{i,j}\in \left\{0,1\right\},\;\forall o_{i},o_{j}\in O\\ \left(\text{b}\right)\overset{n}{\underset{i=1}{\sum }}x_{i,j}=1,\;\forall o_{j}\in O\\ \left(\text{c}\right)\overset{n}{\underset{j=1}{\sum }}x_{i,j}=1,\;\forall o_{i}\in O\\ \left(d\right)c_{i,j}+r_{j}\beta \leq C_{i},\;\forall o_{i},o_{j}\in O\left(T_{i}\right),T_{i}\subseteq T\\ \left(e\right)\overset{n}{\underset{i=1}{\sum }}\overset{n}{\underset{j=1}{\sum }}x_{i,j}\underset{o_{j}\in O}{\sum }f\left(o_{j}\right)\geq \rho . \end{array}$$

There are four steps in Algorithm 2, which are listed as follows:

Step 1: Construct graph *G* by considering set *O* and *S* (Line 1);
Step 2: Initialize the set of ℬ and 𝒬 (Line 2);
Step 3: The following process is invoked when there exists *b* ∈ ℬ is not the primal feasible solution,
  1. Initialize set *𝒥*_*g*_ as *j* when *b*_*j*,*g*_=0,  1 ≤ *j* ≤ *n* (Line 4);
  2. Initialize set ℒ_*g*_ as *i* when ∑_*j*=1_^*n*^*c*_*i*,*j*_*b*_*j*,*g*_ ≤ 0, 1 ≤ *i* ≤ *n* (Line 5);
  3. Find $\tilde{b}$ from *𝒥*_*g*_ satisfying the following equation (Lines 6–9): $\left(c_{\tilde{b}}-\sum_{i=1}^{n}c_{i,r}q_{i,g}|/|\sum_{i\in {ℒ}_{g}}c_{i,r}\right)=\eta =\min_{i\in {ℒ}_{k}}\left(c_{j}-\sum_{i=1}^{n}c_{i,g}q_{i,g}|/|\sum_{i\in {ℒ}_{g}}c_{i,j}\right)$ (6)
  4. Update *b*_*i*,*g*+1_ to 1 when $j=\tilde{b}$ and *b*_*i*,*g*_ otherwise (Lines 10–14);
  5. Update *d*_*i*,*g*+1_ when *i* belongs to set ℒ_*g*_ and *d*_*i*,*g*_ (Lines 15–19);
Step 4: Find the tour *T* through NITSP based on {*z*_*i*_*|* *i*=1,2,…, *n*} (Line 22).

**Theorem 5 .**

CDRS is a polynomial-time approximation algorithm for CDM problem.

**Proof**

Step 1 takes *O*(*n*^2^) time. Steps 2 and 3 take *O*(*n*^2^) time. Step 4 can be finished in polynomial time.

Let opt denote the optimal solution of the CDM problem. The CDRS satisfies the following conditions when *g*=0, *b*_0_=0, and *q*_0_=0.

1. 𝒬_*g*_ is a dual feasible solution;
2. ({*c*}_*e*∈*T*_ − 𝒬_*g*_)ℬ_*g*_=0.

We assume that conditions (1) an (2) are true when *g* ≥ 0.

About condition (1), we find that 𝒬_*g*_ is a dual feasible solution after the coupling hypothesis of condition (1). Thus, *η* is nonnegative. Then, we have *d*_*i*,*g*+1_ ≥ *d*_*i*,*g*_ ≥ 0 when *i* is from 1 to *n*.

According to condition (2), we have *c*_*j*_ − ∑_*j*=1_^*n*^*c*_*j*,*g*_*q*_*j*,*g*_=0 when *j* ∉ ℒ_*g*_. Then, we have ∑_*i*=1_^*n*^*c*_*i*,*g*_*b*_*i*,*g*_=0 for each *i* ∉ *𝒥*_*g*_. So, *c*_*i*,*j*_=0 when *j* ∉ ℒ_*g*_.

Moreover, we have the following equation:

(11) $$\begin{array}{c} c_{j}-\overset{n}{\underset{j=1}{\sum }}c_{j,g}q_{j,g}\\ =c_{j}-\underset{j\notin {ℒ}_{g}}{\sum }c_{j,g}q_{j,g+1}\\ =c_{j}-\underset{j\notin {ℒ}_{g}}{\sum }c_{j,g}q_{j,g}. \end{array}$$

From the process of Lines 6–9, we have

(12) $$\begin{array}{c} \eta \underset{i\in J_{g}}{\sum }c_{i,j}\leq c_{j}-\overset{n}{\underset{i=1}{\sum }}c_{i,j}q_{j,g} \end{array}$$

Furthermore, we have the following equation when *j* ∈ ℒ_*g*_:

(13) $$\begin{array}{c} c_{j}-\overset{n}{\underset{i=1}{\sum }}c_{i,j}q_{j,g+1}\\ =c_{j}-\overset{n}{\underset{i=1}{\sum }}c_{i,j}q_{j,g}-\eta \underset{i\in J_{g}}{\sum }c_{i,j}\geq 0. \end{array}$$

Therefore, 𝒬_*g*+1_ is a dual feasible solution.

For condition (2), we analyze the factor satisfying the inequality ∑_*i*=1_^*n*^*c*_*i*,*j*_*q*_*j*,*g*+1_ ≤ *c*_*j*_. We have the equation ∑_*i*=1_^*n*^*c*_*i*,*j*_*q*_*j*,*g*_ ≤ *c*_*j*_ when *q*_*j*,*g*_ ≤ *q*_*j*,*g*+1_. Based on dual hypothesis, we have *b*_*j*,*g*_=0. In addition, according to the process of Lines 6–9, we also have

(14) $$\begin{array}{c} \overset{n}{\underset{i=1}{\sum }}c_{i,\tilde{b}}q_{j,g+1}\\ =\overset{n}{\underset{i=1}{\sum }}c_{i,\tilde{b}}q_{j,g}+\underset{i\in J_{g}}{\sum }\eta c_{j,g}\\ =\overset{n}{\underset{i=1}{\sum }}c_{i,\tilde{b}}q_{j,g}+c_{\tilde{b}}-\overset{n}{\underset{i=1}{\sum }}c_{i,\tilde{b}}q_{j,g}=c_{\tilde{b}} \end{array}$$

Finally, let *h* be max_1≤*i*≤*n*_∑_*j*=1_^*n*^*c*_*i*,*j*_; we have

(15) $$\begin{array}{c} Q_{g}C{ℬ}_{g}\\ =\overset{n}{\underset{i=1}{\sum }}q_{j,g}\left(\overset{n}{\underset{j=1}{\sum }}c_{i,j}b_{j,g}\right)\\ \leq \overset{n}{\underset{i=1}{\sum }}q_{j,g}\left(\overset{n}{\underset{j=1}{\sum }}c_{i,j}\right)\\ \leq h\overset{n}{\underset{i=1}{\sum }}q_{j,g}\\ =hQ_{g}1_{n}. \end{array}$$

Hence, the process of Lines 2–21 can return an approximation solution.

The NITSP algorithm can find an approximation solution based on set ℬ_*n*_.

Above all, CDRS can find an approximation solution for solving the CDM problem in polynomial time.

## 6. Numerical Experiments

In this section, we conduct extensive simulations to verify the performance of our proposed algorithms with different number of elderly people, battery capacity of drone, initial energy of drone, and number of charging stations.

### 6.1. Simulation Setup and Benchmark

We assume that there are some emergency service request points for the elderly chronic disease deployed in Jiangning Campus of Nanjing Medical University. The elderly people will send the emergency service request at the fixed points. The parameters of drone are from Mavic 2 [22]. In our simulation, we evaluate the total time cost of drone and QoE calculated by the ratio of waiting time to request time. All the simulations were run on a cloud server ECS [23] with 12-core Intel Xeon Platinum 8269CY and 48 GB memory. The other parameter settings of our simulations are listed in Table 2.

1. GT: the Greedy Time (GT) algorithm for solving the DM problem. The algorithm always finds the minimum time cost subtour for the drone greedily starting from *d*_0_ and providing all elderly chronic disease emergency services that satisfy the energy constraint of drone.
2. CGE: the Charging driven Greedy Energy (CGE) algorithm for solving the CDM problem. The algorithm always finds the maximum charging energy subtour for the drone greedily starting from *d*_0_ and providing all elderly chronic disease emergency services that satisfy the energy constraint of drone.

### 6.2. Performance Evaluation

In this subsection, we evaluate the performance of GT, DRS, CGE, and CDRS in the network shown in Tables 3 and 4, which give the locations of emergency service request and charging stations, respectively. The above information is calculated based on the Google map.

Figures 2 and 3 show the impact of number of elderly people on total time cost of GT and DRS, as well as CGE and CDRS, respectively. The results show that DRS and CDRS can reduce 57.38% and 64.06% of total time cost of GT and CGE on average, respectively. This indicates that the proposed algorithms significantly outperform GT and CGE, respectively. This is because the outputs of DRS and CDRS are better than the paths obtained by GT and CGE, respectively.

Figures 4 and 5 show the impact of battery capacity of drone on total time cost of GT and DRS, as well as CGE and CDRS, respectively. The results show that DRS and CDRS can reduce 26.20% and 55.63% of total time cost of GT and CGE on average, respectively. Figures 6 and 7 show the impact of initial energy of drone on total time cost of GT and DRS, as well as CGE and CDRS, respectively. The results show that DRS and CDRS can reduce 21.09% and 56.41% of total time cost of GT and CGE on average, respectively.  Figure 8 shows the impact of number of charging stations on total time cost of CGE and CDRS, respectively. The result shows that CDRS reduces 24.53% of total time cost of CGE on average.

Figures 9 and 10 show the impact of number of elderly people on QoE of GT and DRS, as well as CGE and CDRS, respectively. The results show that DRS and CDRS can increase 55.63% and 89.12% of QoE of GT and CGE on average, respectively. Figures 11 and 12 show the impact of battery capacity of drone on QoE of GT and DRS, as well as CGE and CDRS, respectively. The results show that DRS and CDRS increase 39.09% and 90.75% of QoE of GT and CGE on average, respectively. Figures 13 and 14 show the impact of battery capacity of drone on QoE of GT and DRS, as well as CGE and CDRS, respectively. The results show that DRS and CDRS increase 18.61% and 320.8% of QoE of GT and CGE on average, respectively.  Figure 15 shows the impact of number of charging stations on QoE of CGE and CDRS, respectively. The result shows that CDRS increases 58.31% of QoE of CGE on average.

Overall, DRS and CDRS can not only significantly decrease the total time cost but also increase the QoE through the designed drone assisted emergency service system and its management schemes for elderly chronic disease, respectively.

## 7. Conclusion

In this article, we have designed the drone assisted emergency service system and its management schemes for elderly chronic disease. There is a drone in the area to provide emergency services for chronic diseases, where the drone can be charged by the ground charging stations. Thus, the drone has sufficient energy to provide the emergency service for elderly chronic disease. We have formulated DM problem to minimize the total time cost of drone subject to all elderly chronic disease services which can be guaranteed exactly once by the drone under its energy constraint and proposed the DRS algorithm. To address the limitation of drone, we further formulated the CDM problem to maximize the service utility under the energy constraint of drone and proposed the CDRS algorithm. Through the theoretical analysis and numerical simulation experiments, we demonstrated that DRS and CDRS can decrease the total time cost by 37.61% and increase the QoE by 112.80% through the designed system, respectively.

## Figures and Tables

**Figure 1:** Scenario of drone assisted emergency service management.

**Figure 2:** Total time cost versus number of elderly people.

**Figure 3:** Total time cost versus number of elderly people.

**Figure 4:** Total time cost versus battery capacity of drone.

**Figure 5:** Total time cost versus battery capacity of drone.

**Figure 6:** Total time cost versus initial energy of drone.

**Figure 7:** Total time cost versus initial energy of drone.

**Figure 8:** Total time cost versus number of charging stations.

**Figure 9:** QoE versus number of elderly people.

**Figure 10:** QoE versus number of elderly people.

**Figure 11:** QoE versus battery capacity of drone.

**Figure 12:** QoE versus battery capacity of drone.

**Figure 13:** QoE versus initial energy of drone.

**Figure 14:** QoE versus initial energy of drone.

**Figure 15:** QoE versus number of charging stations.

**Algorithm 1:** DRS.

**Algorithm 2:** CDRS.

**Table 1:** Frequently used notations.

Notation	Description
*O*	Set of *n* elderly people
*r*_*i*_	Time cost of emergency service for the *i*-th elderly chronic disease service
*S*	Set of *m* charging stations
*φ*	Charging power of charging station
*ν*	Flying speed of drone
*σ*_*h*_	Unit hovering energy consumption
*σ*_*f*_	Unit flying energy consumption
*C*_max_	Battery capacity of drone
*d*_0_	Depot for drone
*G*	Emergency service management network
*E*	Set of service segments
*t*_*e*_	Time cost of edge *e* ∈ *E*
*T*	Tour of drone
*β*	Energy consumption of drone providing service
*c*_*e*_	Energy consumption of drone passing through the edge *e*
*𝒞*_*i*_	Residual energy of drone after passing through the edge *e* and completing the *i*-th elderly chronic disease service
*τ*_*k*_	Charging time for drone at charging station *s*_*k*_ ∈ *S*
*T*_*i*_	Drone subtour from the depot to the *i*-th elderly chronic disease service
*O*(*T*_*i*_)	Elderly people serviced by the drone in *T*_*i*_
*S*(*T*_*i*_)	Charging stations visited by the drone in *T*_*i*_

**Table 2:** Parameter settings.

Parameter	Value
*n*	100
*m*	10
*β*	1.5 kW
*φ*	10 kW
*C*_max_	90 Wh
*c*_0_	20 Wh
*r*_*i*_	[1, 5] h

We develop the following benchmark algorithms for comparison:

**Table 3:** Locations of emergency service request.

*i*	Longitude	Latitude
1	31.93433246922838	118.89411397044051
2	31.9385259860767	118.89252407466076
3	31.939684813314848	118.89375307677773
4	31.94081787467635	118.88827567242747
5	31.940289972836105	118.88897362421234
6	31.935422888622234	118.88966481070858
7	31.939230738279367	118.8847133422139
8	31.93754295175468	118.8876962509683
9	31.93555357640813	118.89236190699413
10	31.937852577865236	118.89467251853483

**Table 4:** Locations of charging stations.

*i*	Longitude	Latitude
1	31.933466228677545	118.89180138538082
2	31.93638454072936	118.89252429138394
3	31.93824267776691	118.89280903796829
4	31.938177713559316	118.89275162333368
5	31.937955752188387	118.88729085352668
6	31.93751465301634	118.89001293552754
7	31.942046989944334	118.88759508254144
8	31.935615904900363	118.88827172056612
9	31.934351759640094	118.89139983561418
10	31.93628201571477	118.89392111202842

## Data Availability

The data used to support the findings of this study are included within the article.
